The article "Histopathological features of bone regeneration in a canine segmental ulnar defect model" was retracted in 2016. Reasons: misconduct by an author; plagiarized text; compromised peer review; false authorship.

# Histopathological features of bone regeneration in a canine segmental ulnar defect model

**DOI:** 10.1186/1746-1596-9-59

**Published:** 2014-03-17

**Authors:** Rahim Hobbenaghi, Pariya Mahboob, Siamak Saifzadeh, Javad Javanbakht, Javad Yaghoobi Yeganeh Manesh, Rasool Mortezaee, Seyed Rashid Touni, Ehsan Hosseini, Shahin Aghajanshakeri, Milad Moloudizargari, Soheil Javaherypour

**Affiliations:** 1 Department of Pathology, Faculty of Veterinary Medicine, Urmia University, Urmia, Iran; 2 Graduate, Faculty of Veterinary Medicine, Urmia University, Urmia, Iran; 3 Institute of Health and Biomedical Innovation, Queensland University of Technology, 60 Musk Avenue, Kelvin Grove, Brisbane Qld 4059, Australia; 4 Department of Pathobiology, Faculty of Veterinary Medicine, Tehran University, Tehran, Iran; 5 Gradute of Islamic Azad University of Shahrekord, Faculty of Veterinary Medicine, Shahrekord University, Shahrekord, Iran; 6 Student of Ferdowsi University of Mashhad, Faculty of Veterinary Medicine, Ferdowsi University, Mashahd, Iran; 7 Ph.D Student of Anatomy and Embryology, Faculty of Veterinary Medicine, Urmia University, Urmia, Iran; 8 Faculty of Para Veterinary Medicine, Ilam University, Ilam, Iran; 9 Student of Veterinary Medicine, Faculty of Veterinary Medicine, Urmia University, Urmia, Iran

**Keywords:** Bone defect, Bone regeneration, Vascular bone grafting, Histopathology, Dog

## Abstract

**Background:**

Today, finding an ideal biomaterial to treat the large bone defects, delayed unions and non-unions remains a challenge for orthopaedic surgeions and researchers. Several studies have been carried out on the subject of bone regeneration, each having its own advantages. The present study has been designed in vivo to evaluate the effects of cellular auto-transplantation of tail vertebrae on healing of experimental critical bone defect in a dog model.

**Methods:**

Six indigenous breeds of dog with 32 ± 3.6 kg average weight from both sexes (5 males and 1 female) received bilateral critical-sized ulnar segmental defects. After determining the health condition, divided to 2 groups: The Group I were kept as control I (n = 1) while in Group II (experimental group; n = 5) bioactive bone implants were inserted. The defects were implanted with either autogeneic coccygeal bone grafts in dogs with 3-4 cm diaphyseal defects in the ulna. Defects were stabilized with internal plate fixation, and the control defects were not stabilized. Animals were euthanized at 16 weeks and analyzed by histopathology.

**Results:**

Histological evaluation of this new bone at sixteen weeks postoperatively revealed primarily lamellar bone, with the formation of new cortices and normal-appearing marrow elements. And also reformation cortical compartment and reconstitution of marrow space were observed at the graft-host interface together with graft resorption and necrosis responses. Finally, our data were consistent with the osteoconducting function of the tail autograft.

**Conclusions:**

Our results suggested that the tail vertebrae autograft seemed to be a new source of autogenous cortical bone in order to supporting segmental long bone defects in dogs. Furthermore, cellular autotransplantation was found to be a successful replacement for the tail vertebrae allograft bone at 3-4 cm segmental defects in the canine mid- ulna. Clinical application using graft expanders or bone autotransplantation should be used carefully and requires further investigation.

**Virtual slides:**

The virtual slide(s) for this article can be found here: http://www.diagnosticpathology.diagnomx.eu/vs/2028232688119271.

## Background

Despite the growing knowledge on the mechanisms of fracture healing, delayed healing and non-union formation remain a clinical problem. Delayed unions and especially non-unions do not only result in significant pain and loss of function with subsequent reduction in quality of life, but are also associated with a considerable economic burden to the society [1,2].

Segmental defects and delayed healing of long bone fracture remains a major problem among orthopedic surgeons. Nonunion of the forearm as a result of complex open fracture can result in imbalance in the main anatomical structures, leading to impaired function [3].Furthermore, large bone defects occur mainly as a result of extensive bone loss due to pathological events such as trauma, inflammation [1,2], and surgical treatment of tumours [4,5]. Therefore, the treatment of large bone defects is challenging to orthopedic and reconstructive surgeons. Treatment of bone defects in weight-bearing situations (e.g. limbs) demands the use of a stable construct. Various techniques can be used to bridge defects or regenerate lost bone in these circumstances. Previous studies on the repair of segmental defects have focused on bone matrix substitutes [6-8]. However, these substitute matrices do not perform as well as autograft for several reasons including histochemical responses by the host tissue and a dearth of living cells. Enhancing the osteogenic capabilities of these bone matrix substitutes for the treatment of segmental defects is currently an active area of research. In addition, the use of cytokines and growth factors, such as bone morphogenetic proteins, with and without bone matrix substitutes has great potential for enhancing the bone repair process [9-13] However, few of these studies have been able to demonstrate acceleration of fracture healing. In human, the formation of new blood vessels (vasculogenesis or angiogenesis) plays an important role during osteogenesis and bone healing [14]. These observations are in accordance with those of a previous study that suggested that the Kombucha fungus accelerates the healing quality [15,16]. In fracture repair [17,18] and distraction osteogenesis [19,20], vascular changes precede bone formation. In the rat ulnar fracture model, the spatial pattern of maximal vascular changes along the ulna is identical to the pattern of woven bone formation [21].

Bone grafts are the most common methods for treating various types of bone defects, nonunions, delayed unions, osteomyelitis and large bone defects. Different bone grafts are include autograft,isograft, allograft, alloimplant and xenograft. Bone grafting is of commonly surgical indications of small animals bone fractures, mostly applied to making bridge for huge bone defects or repairing of long bone [22,23]. Autogenous bone graft has been considered the gold standard for bone-repairing procedures as it contains the triggering ingredients necessary for bone formation in cases of bone defect. However, the availability of auto-graft bone is limited, and the harvesting of autograft bone causes morbidity at the donor site. Allografts have become common alternatives to autografts [24-26].

Animal models in bone repair research include representations of normal fracture healing, segmental bone defects, and fracture non-unions in regular healing processes are compromised without presence of a critical-sized defect site [27]. Recently, the use of dogs as experimental models has significantly decreased mainly due to ethical issues and approximately 9% of articles published in leading orthopaedic and musculoskeletal journals described dogs as animal models for fracture healing research [28].

The aim of this research is to evaluating pathological caudal vertebrae functions in experimental defects of dog ulna bone, and introducing such method as an applicable method in small animals’ orthopedics.

## Methods

### Ethics statement

All experiments described in this study were performed in full accordance with the guidelines for animal experiments released by the National Institute of Animal Health. This study was approved by the Animal Ethics Committee at Urmia University (Ethics code permit no. TU2013-1-11-007Y). The animals were placed in shade, in standard conditions, water ad libitum, and without restriction of movement according to the guidelines of the Institutional Animal Ethical Committee of the Urmia University of Animal Science, Iran. Surgery was performed under aseptic conditions and sedation by injection of xylazine hydrochloride (0.05 mg/kg) followed by 2% lignocaine hydrochloride (Table 1). The blood samples were collected for routine tests from cephalic vein one week prior to surgery. Furthermore, anti-parasitic drugs administered (Praziquantel, Ivermectin, Levamisole), and the rabies vaccine injected to each dog (1 cc), the diet was same and fed manually. The water was easily accessible as well.

**Table 1:** Characterization of experimental dog model

**Group**	**Sex**	**Breed**	**Weight**
Test	Female	Native	28
Test	Male	Native	32
Test	Male	Native	35
Test	Male	Native	30
Test	Male	Native	32
Control	Male	Native	34
The average weight (kg)			32 ± 3.6

### History and clinical examination

In the present study, six indigenous breeds of dog with 32 ± 3.6 kg average weight from both sexes (5 males and 1 female) examined. After determining the health condition, divided to 2 groups: The Group I were kept as control (1case, Control group) while in Group II (5 cases, Test group), bioactive bone implant were inserted (Table 1).

### Anesthesia

The anesthetic for each of the cases was xylazine HCl (Alfazine® 2%, Alfasan/Egevet, Iran) (1 mg/kg, IM) followed by thiopental Na (Pentothal Na® 1 g, Abbott, UK) (15 mg/kg, IV) and ketamine HCl (Alfamine® 10%, Alfasan/Egevet, Iran) (10 mg/kg, IM) in dogs respectively. General anesthesia was maintained with 2% isoflurane (Forane® Abbott, UK). Respiration was maintained with mechanic ventilation (15 ml/kg tidal volume, respiration rate 15/min and 25 cm H_2_ O airway pressure). All of the cases were monitored with ECG, a pulse-oximeter and a capnograph.

### Surgery technique

In this assessment each dog had 2 operations: 1) Cosmetic caudectomy and caudal vertebrae removing for bone replacement. Cosmetic caudectomy carried out as described in Fossum et al. 2002 [29]. Subsequently, soft tissues such as skin and muscles dissected and vertebral bones disarticulated. So the 6^th^ and 7^th^ bone removed. The cartilage surface removed by scalpel and the bone processes reformed by bone rongeur then longitudinal canal made in vertebrae bone medulla by a bone 3 mm pin drill (Figure 1A and B), and the vertebrae length measured and kept in a moist tampon. 2) Making bone defect in left ulna and caudal vertebrae bone replacement. A cutaneous incision (10 cm) created over antebrachium on ulna through caudolateral approach. After dissection of subcutaneous and muscular tissues, a cylindrical defect made by gigli wire similar to caudal vertebrae size in the middle of ulna (Figure 1C and D).

**Figure 1:** ***Gross morphological *characteristics of cosmetic caudectomy and caudal vertebrae removing together with making bone defect in left ulna and caudal vertebrae for bone replacement; A: Indicates the caudal vertebrae processes reforming by ronguer forceps. B**: Represents that a longitudinal canal made in a fixed vertebra by a 3 mm pin drill and a bone forceps. **C**: Shows that a defect as long as the caudal vertebrae created in ulna bone by gigli wire. **D**: The created defect in ulna bone is observable. **E**: The caudal vertebrae replacement in the ulnar bone defect.

Subsequently, the caudal vertebrae replaced and fixed in defect by orthopedic drill with a 3 mm medullary pin through Normograde technique which entered from olecranon process and the cylindrical bone replaced by bone forceps (Figure 1E). Then the rotating bone pin passed through caudal vertebra medullary canal and entered ulna bone that the pin moving direction was toward distal part. Upon proper fixation the additional part of pin in olecranon process has resected, and the cutaneous incision sutured by non-absorbable suture with cruciate pattern. In control group the cosmetic caudectomy was similar to test group, but the defect did not filled with bone graft and the upper and lower parts fixed together by a 3 mm intramedullary pin.

Postoperatively, each case received additional care. Fluid infusion, ampicillin sulbactam (20 mg/kg, i.v.) (Combisid® 1 mg, Sina, Tehran) and pethidine HCl (5 mg/kg, i.v.), (Aldolan® ampoule 100 mg, Heydari Pharmacy, Tehran) were administered.

### Histological study

The implanted bones were collected from the animals at day 120 postoperatively. The sections were cut (3–4 mm thick) using hacksaw including both normal and implanted area of bone. The bone pieces were washed thoroughly with normal saline and were fixed in 10% formalin for 15 days. Subsequently bones were decalcified in Goodling and Stewart’s fluid containing formic acid 15 ml, formalin 5 ml and distilled water 80 ml solution and it was stirred daily and changed once in three days. The sections were checked regularly for the status of decalcification. They were considered as completely decalcified when sections became flexible, transparent and easily penetrable by pin. The decalcified tissues were processed in a routine manner and 4-5 μm sections were cut and stained with Haematoxylin and Eosin. The stained sections were observed for status of the bone implants and cellular response of host bone to the implants.

## Results

### Finding control group

Histologically, extensive fibrotic texture was obvious in the newly organized tissue, and contained abundant collagen fibers, somehow such fibrotic tissue could connect to bone, and small immature bone Lamellas created, but nearly all of defect spaces occupied by fibrotic tissue (Figure 2A). In parallel, small bone Lamellae made by host compact bone tissue. Moreover, two small bone Lamellae foci created amongst fibrotic tissue irregularly (Figure 2B).

**Figure 2:** **Hitopathological evaluation of on the autotransplantation of tail vertebrae for segmental bone defect reconstruction in dogs; A: It demonstrates the defect filling by dense connective tissue and no cortex formation in control group.** (H&E, 48×), **B**: Shows the partial, small and irregular bone lamellar formation at sides of control group defect. (H&E, 150×), **C**: It indicates the compact bone formation at the lower cortex and continuous osteogenesis at the upper side. Furthermore, the necrotic residues of autograft bone which has been lysing are visible, and the the middle hole filled by mesenchymal tissue. (H&E, 48×), **D**: Shows the hyperchromaticmesenchymal and osteoclast cells in autograft vertebrae holes of test group. (H&E, 600×), **E**: Represents the impaction of some caudal vertebrae holes by granulation tissue which contains new vessels. (H&E, 150×), **F**: Shows the osteolysis and new bone Lamellar formation of caudal vertebrae autograft residues. (H&E, 150×), **G**: Demonstrates the new bone lamellar formation by periosteum in test group. (H&E, 200×), **H**: Shows the test group intramembranous ossification. (H&E, 600×), **I**: indicates the test group endochondral ossification. (H&E, 600×).

### Experimental group findings

The caudal vertebrae autograft fusion with host bone was 100%, somehow such tissue was entirely osseous and the autograft bone was aligned with the host bone along with new arrays created in them. The graft bone is able to be in harmony with host bone through producing holes and converting them to woven bone, making new Lamellas. At lateral surfaces of autograft at one side created compact bone with cortex, however, no soft tissue (Fibrotic or regenerative mesenchyme tissue) exist at this side, furthermore roughly 100% of bone Lamellae converted to compact bone, whereas at another side bone Lamellas and trabecules formed through numerous regenerations of mesenchymal tissue that partially formed compact bone at junction zones.

Additionally, the medulla of autograft vertebrae developed osteolysis, and its bone Lamellas indicated necrosis process, somewhat remained among bone Lamellas and undergo lysing autograft vertebrae. Hyperchromic mesenchymal cells in holes were observable that regularly aligned in the vicinity of the bone Lamellas, forming new Lamellas which osteoclasts observed at holes as well (Figure 2C and D).

However, some holes impacted by granulation tissue (Figure 2E). The autografting and colourless bone Lamellas connected to newly created live compact Lamellas of host at all dimensions (above and sides) and no differentiation could be diagnosed between them (Except the color and texture, the autograft was hypochromic and undergo lysing) (Figure 2F). The osteogenesis process in depth of autograft was visible at lateral surfaces even the newly lysed bone Lamellas was regenerating. The internal formed Lamellas which directed to upper and lower of the cortex induced to augment bone compaction. At the outer layer of cortex, the new bone Lamellas created by periosteum as well (Figure 2G).

In addition to osteogenesis at depth tissue and gradual compaction toward cortex, at the outer portion the periosteum cortex has developed osteogenesis (Intramembranous ossification) (Figure 2H), and another figure presents a chondral tissue focus that forms bone Lamellas (Endochondral ossification) (Figure 2I).

## Discussion

Bone grafts are often necessary to provide support, fill voids and enhance biologic repair of skeletal defects. Strategies for the development of biological substitutes capable of mimicking the homeostasis are based on a better understanding of the basic events in the healing of the fractures. The biological approach aims to provide the key components which play a pivotal role in the repair of the bone [28,30].

The percent study indicated that usage of 6^th^ and 7^th^ caudal vertebrae as an autograft in critical-sized segmental defect of dogs ulna bone induced remarkable healing after 16 weeks, and was able to reproduce the bone natural uniformity. Evaluation of bone healing by dog ulnar segmental defect model reported by Keg in 1934 for the first time, meanwhile such model would be beneficial for bone grafts and bone graft replacers as produces the least complications [31]. The only report of using caudal vertebrae for dog bone fracture healing published by Blake in 1967, pertaining to a two-year old Terrier with a 2.5 months nonunion tibial fracture [32].

The histology is the best method for bone defect healing evaluation. In present study bone integration indicates new bone formation between host and caudal vertebrae autograft histologically. The caudal autograft with host bone was integrated, somehow no fibrotic tissue observed, and considerable callus between them was visible that produced integration during 16 weeks.

Clinically, in all the surgically created defect areas, the implants were well placed, well accepted and tolerated by the animals, causing no serious inflammation in the surrounding tissue. Healing was uneventful in all animals and there was no evidence of rejection of implant in any case which corroborated with the findings of Holmes et al. (1986) [33]. Lameness disappeared gradually, which suggest that even the resulted mild inflammation was subsided and fracture was getting stable. This finding was in agreement with the observations of ulnar fracture in dog by Shukla (1989) and in rabbit by Singh (2000) [34,35]. In the present study no foreign body response or toxicity was elicited and hence the implant was accepted as a suitable alternative bone graft to fill the defect.

In Group II, the histological section showed well developed lamellar bone containing fair number of havarsian canals and evidence of fair number of blood vessels with marrow element in medullary space. These results are suggesting a process of mesenchymal cells recruitment of surrounding tissues and their subsequent transformation to bone forming cells [36]. The bioactive glass blocks showed osteoconductive and osteointegration properties, as documented in the present study by the close contact between the material and newly formed bone, as well as bone growth around and inside of them. The histological material also showed areas with osteoid tissue (bone tissue being formed), which would call for a longer time for bone maturation and complete resorption of the material with bone replacement. Similar findings are also observed by Macedo et al. using bioactive glass in rat tibias [37]. No bioactive glass material was seen at any region suggesting quick reabsorption of this material than hydroxyapatite, thus allowing a much more precocious new bone formation in the repair of bone defects [36,37]. Besides, the material could not be seen in the present study might be due to the fact that they were completely incorporated into the newly formed bone tissue which is in conformity with the observations of Oonishi et al. (1997) [38].

On the other hand, the periostium vessels contain sources of vascular pericytes that its pluripotential cells are able change to osteoblasts [39]. The osteogenesis at the outer layer where has the highest Lamellas density indicates that the bone growth producing factors from autograft caused host periostum stimulation to osteogenesis. The test group compared to control group showed that no osteogenesis and periosteum development occurred at defect region. So the presence of caudal vertebrae autograft plays the osteoinduction role for host tissue and causes new bone formation. The periostum cells hyperplasia and their incorporation in osteogenesis can be attributed to new bone Lamellas conducting roles that provide conditions to form new bone Lamellas. As mentioned, in undergo lysing autograft Lamellas the osteogenesis cells and other medullary cells exist actively and they are producing new Lamellas, however. Nevertheless, the vanishing autograft Lamellas are align with the host bone Lamellas and connected to each other. Such process indicates new bone Lamellas growth exactly from caudal vertebrae autograft [39].

Furthermore, this study demonstrated that the interface was bridged by cortical bone that probably made through directly defect filling by woven trabecular bone, inducing to caudal vertebrae autograft replacing during 16 weeks, also in this research some holes impacted by meduallary live cells (Bone marrow cells and osteoclasts) at autograft junction site that such cells were lysing the Lamellas and helped regeneration. Additionally, the periosteum cells of the host ulnar bone completely covered caudal vertebral autograft and was hyperplastic as such cells could produce new bone Lamellas on compact bones and cortex, originates from cambium layer function, and contains osteoprogenitor cells that enjoy osteoblasts phenotype genetically [39].

The rapid progression of bone graft research and the great number of novel developments must be supported by systematic assessment based on clinical practicability and experience, the knowledge of basic biological principles, medical necessity, and commercial practicality [40]. From our literature observation, it can be concluded, that in a majority of the mentioned studies, follow-up periods, which in most cases don’t exceed 4-5 months, are not suitable to evaluate long-term effects of bone substitutes and scaffolds on bone regeneration and remodelling, and to determine in vivo resorption kinetics of the respective biomaterial.

## Conclusions

In summary, we found that use of a cancellous autograft approach and bilateral internal plate fixation was efficacious for the treatment of segmental ulnar fractures. Complications were minimal and healing satisfactory. We advocate the use of this approach for repair of segmental ulnar fractures. Furthermore, more studies are needed, for longer periods of time, using other types of autotransplantation of tail vertebrae in order to find the optimal materials, which can serve as segmental ulnar defect for guided bone regeneration.

## Competing interests

The authors declare that they have no competing interests.

## Authors’ contributions

RH, PM and SS participated in the histopathological evaluation, performed the literature review, acquired photomicrographs and drafted the manuscript and gave the final histopathological diagnosis and designed and carried out all the experiments and, participated in the design of the study, performed the statistical analysis .JJ and EH are the principal investigator of the laboratory in which the research was performed and contributed to the interpretation of the data and writing of the manuscript. JYYM, RM, SRT, SHA, MM and SJ edited the manuscript and made required changes and wrote the manuscript. All authors have read and approved the final manuscript.
